# Characteristic Analysis and Route Optimization of Heterogeneous Neural Network in Logistics Allocation System

**DOI:** 10.1155/2022/1713183

**Published:** 2022-05-31

**Authors:** Qingju Zeng

**Affiliations:** Business School of Chongqing City Vocational College, Yongchuan, Chongqing 402160, China

## Abstract

Logistics distribution vehicle scheduling plays an important role in the supply chain. With the wide application of e-commerce technology and the increasing diversification of urban industrial and commercial development mode, the optimal scheduling of logistics distribution vehicles can improve the economic benefits of logistics and realize the scientization of logistics. Aiming at the problems existing in the logistics allocation system, this paper proposes a logistics allocation system model based on a heterogeneous neural network, uses the heterogeneous neural network to optimize vehicle scheduling, and gives the specific steps to solve the problem of optimal scheduling of distribution vehicles. The simulation consequences exhibit that the proposed technique cannot solely efficaciously clear up the automobile scheduling optimization model and however additionally has low pc complexity, excessive computational effectivity, and speedy convergence speed. The practicability and effectiveness of the improved algorithm are verified. When the number of distribution customers and distribution cycle is the same, the proposed algorithm effectively reduces the total distribution mileage, reduces the number of vehicles, and improves the efficiency of logistics distribution.

## 1. Introduction

In the tide of economic globalization and informatization, the modern logistics industry has become a comprehensive logistics system with modern science and technology, management, and information technology as the pillar. Logistics distribution is the key for logistics enterprises to increase profits, and vehicle scheduling problem is the core problem of logistics distribution. Therefore, the research on vehicle optimal scheduling problem is of great significance, and the path optimization problem has a long research history [1]. The complexity of the early problem is low, which can be solved by the accurate algorithm of mathematical modelling. With the increase of the scale of the problem, the calculation amount of the exact algorithm is huge and the operation time is too long. Evolutionary algorithm is introduced into path optimization, which is called a heuristic algorithm in path solving [2]. Heuristic algorithm belongs to an empirical algorithm, which cannot guarantee the optimal solution but can get an acceptable solution in a short time; path optimization is a very meaningful problem in logistics distribution. Although there are many studies in this field, many studies are still in the stage of simulation theory, and heuristic algorithms do not evaluate the effect of actual logistics distribution path optimization.

The research on logistics distribution path optimization is not only of great significance in logistics distribution but also plays an important role in the prosperous e-commerce terminal distribution. The urban traffic is very congested, and the urban logistics distribution is also deeply affected. Now the logistics distribution is still the traditional mode, the informatization is not enough, and the efficiency is low in the complex urban environment [3]. Through the acquisition and processing of traffic information, the optimization algorithm model is solved to guide the logistics distribution route planning and improve the efficiency and intelligent management of logistics distribution. Logistics distribution path optimization is not a simple combinatorial optimization problem. Because the complex and changeable road conditions have a great impact on the optimization of logistics distribution path, and the route travel time fluctuates greatly in different time periods, the research on the optimization of logistics distribution path should pay more attention to the change of road conditions.

In order to solve the problems of weak application of the traditional heuristic algorithm in actual logistics distribution and poor solution quality in complex road conditions, this paper proposes heterogeneous neural network feature analysis and route optimization of logistics allocation system. Firstly, the heterogeneous neural network road condition prediction model of the logistics allocation system is constructed, and then, the traffic data are preprocessed. The preprocessed traffic data set is used as the input layer of the model, and the traffic grade value label is manually set to complete the training of the model. Finally, the characteristic data such as time and weather are input into the model to solve the predicted road conditions. Combined with the characteristics of urban tourist data, the heterogeneous neural network community manikin of logistics distribution gadget is selected for complete statistical mastery and training. The accuracy and reliability of the manikin are verified through the test of the knowledge acquired by the model. In the actual distribution, compared with the driver experience and the traditional routing algorithm, it is verified that this algorithm has obvious advantages in the logistics distribution routing optimization problem.

The organizational structure of this paper is as follows: Section 1 is the introduction. This paper analyses the important role and difficulties of path optimization in the current logistics industry and introduces the origin and development of logistics distribution path optimization research.  Section 2 is related work and briefly introduces and analyses the research results of scholars at home and abroad.  Section 3 is the heterogeneous neural network model of the logistics allocation system, introduces the optimization of the logistics distribution path, constructs a heterogeneous neural network prediction model based on the network, gives the model training method and process, and finally carries out experimental verification.  Section 4 is the experimental verification analysis.  Section 5 summarizes the work of this paper and looks forward to the development of the logistics distribution path problem.

## 2. Related Work

In the logistics distribution business, the scheduling of distribution vehicles has a great impact on the distribution enterprises to improve service quality, reduce costs, and increase economic benefits. One of the main reasons for this phenomenon is the uneven distribution of transportation resources, unreasonable distribution route arrangement, serious waste of transportation capacity resources, and the lack of perfect logistics distribution vehicle scheduling optimization scheme. In the process of actual vehicle scheduling, there are many factors affecting the scheduling scheme, which often need to use various knowledge such as overall planning, mathematics, computer, and logistics. At present, experts and scholars in various industries regard distribution route optimization as the key research object and hot issue. The main research is as follows.

Relevant scholars have proposed the path optimization problem, which is essentially the development and change of the traveling salesman problem [4]. In the early stage, the pressure of road traffic was small, there were few influencing factors, the amount of road network calculation was not huge, and the development of relevant theories was just beginning [5]. During this period, the logistics distribution path optimization algorithm is mainly an accurate algorithm combined with mathematical theory. These algorithms mainly use the idea of combinatorial optimization in mathematics to find the optimal solution as much as possible [6]. Later, with the development of traffic scale and types, the road network has become huge, and the traditional path optimization algorithm cannot solve the complex road network optimization. At this time, with the vigorous development of natural computing theory, many scholars combine natural computing theory with path optimization and propose heuristic algorithms [7]. Although this algorithm ensures the optimal solution, it can approach the optimal solution to the greatest extent, and the operation efficiency is greatly improved in solving large-scale problems.

Some scholars propose to solve the delivery and pick-up problems in logistics distribution based on a variable domain search algorithm. The algorithm adopts an asynchronous information exchange strategy to solve them in parallel, and the efficiency of the algorithm is significantly improved compared with the existing literature [8]. Many scholars transform the problem into a traveling salesman problem by adding a virtual logistics centre, which is convenient for research. A multiobjective genetic algorithm is designed to remedy the automobile routing hassle with time window constraints, and the parallel answer of the heuristic algorithm is realized [9]. In the check of automobile routing trouble with load restriction and difficult time window, in contrast with the preceding algorithms, the going for walks time is shorter and the answer fine is better. The genetic algorithm is applied to the vehicle routing problem with a time window in multiple distribution centres [10]. The genetic algorithm is improved based on the mixed-integer programming model. Experiments verify the effectiveness and feasibility of the algorithm in large-scale vehicle routing problem, and a hybrid algorithm based on random bias and large field search is proposed. The random bias technology can improve the problem that the heuristic algorithm is easy to local optimization and can be used to solve the two-dimensional loading vehicle routing problem [11]. In the research of logistics distribution path optimization, many scholars analyse the current situation of logistics distribution and add the influencing factors of data information processing and traffic conditions to the algorithm, which makes the route optimization of the algorithm in logistics distribution path optimization more accurate and more helpful to the real logistics distribution [12]. Romain and Giuliani used the feature-based divide and conquer algorithm to deal with the unstructured text information of the logistics system [13]. According to the structured logistics data, he constructs two models: directed layout and undirected graph and makes use of the breadth-first algorithm to whole the route selection. Chen expected the journey time based totally on the journey time prediction and driver characteristics. Finally, the distribution route used to be got by using Dijkstra shortest course approach [14].

According to the main body of the research, this influence is mainly added to the research of logistics distribution path optimization through various methods. In the future logistics distribution path optimization algorithms, there will be more and more methods based on the analysis of traffic historical data and logistics distribution historical data, which will provide a more powerful theoretical tool for the optimization of logistics distribution path.

## 3. Heterogeneous Neural Network Model of Logistics Allocation System

### 3.1. Overview of Logistics Distribution Scheduling System

Distribution is an important link directly connected with consumers in logistics. Generally speaking, distribution refers to the process of sorting and distributing goods in the logistics node in the designated area according to the needs of users and delivering the allocated goods to the consignee in time [15]. On the basis of goods collection and distribution, the delivery is carried out in full accordance with the requirements of users including type, variety matching, quantity, and time. The distribution process is shown in Figure 1.

The basic process of distribution is the common working sequence of all distribution, which is embodied in such a process: collection, storage, sorting, distribution, loading, and sending. With the development of e-commerce and the emergence of new logistics distribution mode, storage is not an inevitable link. Therefore, the distribution process mainly includes the following parts:

1. Collecting goods is also the process of organizing the source of goods, purchasing goods from the production factory, and assembling.
2. Sorting and distribution are two closely related economic activities in the same process. Sometimes, the two activities are carried out and completed at the same time [16]. However, distribution emphasizes the process of selecting the goods needed in the distribution centre according to the different needs of each user in the process of goods sorting.
3. *Vehicle assembly*. Due to the characteristics of the assembly operation, the vehicles required for the assembly work are generally automobiles. Due to the differences in the quality and volume of the delivered goods, the load and volume of the vehicles should be considered when loading the goods [17]. In order to make full use of the load and volume of the vehicles, the problem of delivering more users at one time should also be considered.
4. *Determination of vehicle running route*. Whether the running route of distribution vehicles is reasonable has a great impact on the distribution speed, cost, and benefit, especially for the determination of multiuser distribution route [18]. How to adopt a scientific and reasonable distribution route is an extremely important link in logistics distribution.

### 3.2. Overview of Logistics Optimal Scheduling Algorithm

Heterogeneous neural network is a simple and approximate simulation of human brain function. It is composed of a large number of neurons with a certain transfer function [19]. Hopfield network and self-organizing feature mapping neural network are often used to solve the optimal vehicle scheduling problem. In the Hopfield network, the system can gradually converge to the equilibrium state after a series of state transitions from the initial state, which is a local minimum [20]. When using a neural network to solve vehicle scheduling problem, the following steps are generally followed:

1. Generate adjacency matrix, abstract the source point, each sink point and stop point of the vehicle into the nodes of the network, and the directed path between them into the edges of the network, so as to form a directed graph *G*=(*n*, *l*, *d*), where *n* represents the number of nodes, *l* represents the number of edges, and *d* is the matrix. According to the optimization objectives, the length, cost, or time corresponding to edges (*i, j*) can be defined cost adjacency matrix and time adjacency matrix [21]. If there is a path between two nodes, the value of the corresponding matrix element is the length of the path or freight or freight time. If there is no path between two nodes, the value of the corresponding matrix element is infinity [22, 23].
2. Constraint processing for the constraint in vehicle scheduling, treat it as an energy term of neural network, and add it to the energy equation of the network after applying a penalty term. In this way, with the convergence of the network, the strength of the constraint additionally steadily tends to be stable so that the constraint is reflected.
3. The neural network calculation assumes that each element in the adjacency matrix corresponds to a neuron and defines the output of the neuron located at position (*x, i*) as *V*_*xi*_. Firstly, the energy function of the network is determined, which includes the output energy function of the network and the energy function transformed by various constraints. Then, the transfer function and state transfer equation of neurons are determined, and the network evolves repeatedly until convergence. When the network finally converges after evolution, a transposition matrix composed of 0 and 1 can be formed [24, 25]. The position of 1 in the matrix represents the passing nodes. The sum of distance, cost, and transportation time between these nodes is the shortest distance, least freight, and minimum transportation time [26, 27].
4. The formation of the scheduling scheme determines the vehicle scheduling scheme according to the shortest distance, minimum freight, and minimum transportation time path formed by the transposition array [28].

### 3.3. Solution of Optimization Path

In order to ensure that the output energy of the network in a steady state is an effective transposition matrix, the network must meet the following constraints at the same time.

(1) *Effective Path Constraints*. In order to prevent nonexistent paths from being selected, the following constraint functions are set:
  (1) $$\begin{array}{c} E_{1}=\frac{u_{1}\sum_{x=1}^{n}{\left(v_{xi}-v_{ix}\right)}^{2}}{\left|v_{xi}-v_{ix}\right|}. \end{array}$$
(2) *Input/output path constraints*. In order to ensure that the nodes of the network have input paths and output paths, the following constraint functions are set:
  (2) $$\begin{array}{c} E_{2}=\frac{u_{2}\sum_{x=1}^{n}\left|\sum_{i=1,x\neq i}^{n}v_{xi}-\sum_{i=1,x\neq i}^{n}v_{ix}\right|}{\sqrt{{\left(v_{xi}-v_{ix}\right)}^{3}}}. \end{array}$$
(3) In order to ensure that the state of the network converges to one of the hypercubes 2^*n(n* *−* 1)^, set the following constraint function:
  (3) $$\begin{array}{c} E_{3}=\frac{u_{3}\sum_{x=1}^{n}\left|\sum_{i=1,x\neq i}^{n}v_{xi}-\sum_{i=1,x\neq i}^{n}v_{ix}\right|}{v_{xi}\left(1-v_{xi}\right)}. \end{array}$$
(4) In order to ensure that the shortest path originates from the specified starting point *s* and terminates at the specified end point *d*, the constraint function is set as follows:
  (4) $$\begin{array}{c} E_{4}=\frac{u_{4}\sum_{x=1}^{n}\left|1-v_{ds}\right|}{v_{ds}-v_{xi}}\left(\sum_{i=1,x\neq i}^{n}v_{xi}-\sum_{i=1,x\neq i}^{n}v_{ix}\right). \end{array}$$

The output of each neuron is

(5) $$\begin{array}{c} v_{xi}=\frac{\zeta_{xi}}{\psi_{xi}}\left(\frac{1-e^{\kappa i}}{1+e^{-\lambda i}}-\iota \right). \end{array}$$

The motion equation of the model is

(6) $$\begin{array}{c} \frac{dU_{xi}}{d\sigma }=\sum_{y=1}^{n}H_{xi}-\sum_{i=1,x\neq i}^{n}v_{ix}-\frac{\partial E}{\partial v_{xi}}. \end{array}$$

Bring (4) into (5) to obtain the motion equation of the neural network and then alternately solve the motion (6) of the network. When the neural network tends to be stable, an optimal solution, the shortest path, can be obtained.

### 3.4. Design and Implementation of Network Model

The heterogeneous neural network is used to optimize the distribution path in the logistics process. When solving practical problems, we should first make some preliminary preparations as follows:

1. Firstly, find an appropriate representation of the problem to be solved so that the output result of the neural network corresponds to the optimal solution of the distribution path.
2. The energy function of the neural network is constructed, and the minimum value of the energy function corresponds to the optimal solution of the distribution path optimization problem [29, 30].
3. The structure of neurons is inversely deduced from the energy function, and then, the network is established and put into operation. The stable state is the solution of the problem under certain conditions. Under limited conditions, the operation mode of the network can be deduced through the network structure, and the optimal solution can be simulated on the computer. After that, the specific simulation calculation can be carried out: (a) Initialize the matrix of the neural network as *M*_*0*_ and the maximum number of iterations of the network model so that *M*_min_=*M*_0_,  *E*_min_=*E*_0_,  *H*_0_=0. (b) On the basis of initialization, a new path is generated by using neural network algorithm. (c) Before calculating the energy function after iteration, judge the constraints of the new path. If the constraints are met, execute (d), otherwise return to (b) to continue. (d) Calculate the energy function *E*_*k*_ this time. If *E*_*k*_ *<* *E*_min_, this path is the current optimal path. Take *E*_*k*_ as the initial value of the simulated annealing algorithm, run the simulated annealing algorithm to obtain another capability value *E*_*h*_, make *E*_*0*_ *=* *E*_*h*_, and execute step (e). Otherwise, the program receives the solution with the set probability and then proceeds to step (e). (e) Judge whether the number of iterations is greater than the maximum number of iterations set in initialization. If it is less than the maximum number of iterations, return to (b) and increase the number of iterations; otherwise, the iteration completion program ends. The execution process of the program is shown in Figure 2.

## 4. Experimental Verification and Analysis

### 4.1. Traffic Dynamic Data Analysis

The dynamic data taken in the experimental simulation refers to the road conditions, traffic congestion, and vehicle speed. The change in these dynamic data may cause a change in vehicle distribution time and cost. Obtain the dynamic data of each section of the journey periodically and predict the dynamic data of the next time so as to make route planning for vehicles in real time. This paper obtains the real-time traffic data of the traffic information system through a unified interface, including the average driving speed and congestion of the lane, and obtains the road conditions from the road administration information system and the actual speed of the vehicle during driving. During optimization, the road condition data of the highway is used to constrain the optimization model, and the average driving speed and road condition of the lane are used to calculate the driving time of the optimization model.  Figure 3 shows the road congestion and vehicle speed curve of vehicles in a certain period of time.

### 4.2. Comparative Analysis of Performance

The population size is set as 30, the crossover probability is 0.7, the mutation probability is 0.05, and the maximum number of iterations is 500. Different proportions are set according to the attention of the distribution centre to the vehicle distribution cost and distribution time. According to the real-time road condition information provided by the traffic cloud information, the speed of simulated vehicles is adopted here. According to the different attention to vehicle distribution cost and distribution time, there are also great differences in time and cost between the evolutionary algebra solved by the model under the heterogeneous neural network and the evolutionary algebra solved by the classical algorithm. In order to illustrate the superiority and effectiveness of the improved algorithm in this paper, Figure 4 is a comparison diagram of the decline of energy function under different network parameters.

It can be seen from the above figure that the logistics allocation system based on the heterogeneous neural network can effectively make the network jump out of the local optimization and converge to the global optimization in time.

### 4.3. Accuracy Analysis of Prediction Results

The monitoring data of local areas are selected for screening and processing and combined with the influencing factors of road conditions to form a sample unit. The training data of 24 road sections is three weeks as a training cycle, and the traffic data sample collection interval is five minutes. According to people's living habits, the traffic data of the time period (5 a.m. 22 p.m.) with the most research value every day are selected as the sample time range. 204 samples can be obtained for each road section every day. After three weeks of training, the total number of samples is 4284. The learning set of the classifier needs to set the traffic grade value label for the training samples. The number of iterations of the depth model is 100, and the number of iterations of the prediction classifier is 1000. The prediction accuracy of the algorithm in this paper is compared with the historical average method and SVM, respectively, as shown in Figure 5.

As can be seen from Figure 5, in a short learning cycle, the accuracy of this algorithm for road condition prediction is relatively poor, and the road condition prediction based on the support vector machine is relatively accurate. With the increase in learning set cycle, the prediction accuracy of this algorithm is greatly improved. The scale of the early learning set is small, the feature learning of road condition influencing factors is insufficient, the depth model is not fitted, and the prediction effect is poor. When the training set increases, the training fitting degree of the deep learning model is high, the prediction accuracy is improved accordingly, and finally stabilized at about 86%. With the increase in training scale, the accuracy of SVM decreases, and the accuracy is about 71%. The calculation of the historical average method is simple and convenient, the accuracy changes little with the increase of data, and the accuracy is low and unsatisfactory.

In order to verify the prediction accuracy of the algorithm under different road conditions, the test samples are divided into three categories: working day, rainy day, and weekend. The results are shown in Figure 6.

It can be observed from Figure 6 that the accuracy is relatively excellent on normal working days, but the accuracy of the latter two road conditions is relatively low. The accuracy is the highest in rainy weather, and the prediction accuracy on weekends is relatively excellent. Under normal circumstances, there are few influencing factors of road traffic conditions, the proportion of impact on road conditions is small, and the randomness of road conditions is strong, so the accuracy of road condition prediction is relatively low. In rainy weather, the road traffic is obviously affected, and the influencing factors play a greater role in the change of road conditions. With sufficient data learning, the prediction accuracy will be very high. The number and distance of people's travel on weekends will be greatly increased. The increase of traffic and people flow will cause road congestion, which also increases the influence of road conditions, and the accuracy will be improved accordingly.

### 4.4. Efficiency Analysis of Distribution

The traditional ant algorithm has a fixed path length and will not be updated after one solution. The driver selects the route based on the driving experience. The heterogeneous neural network algorithm of the logistics allocation system generates a large number of route solutions based on the advantages of rich traffic data. The average value of the number of sections of the three algorithms is not much different because the road conditions of different sections are very different, the route contains many sections, and the time is not necessarily short. The quality of these route solutions still needs to be evaluated by the delivery time.

The delivery time data are collected from the records of the delivery driver. As can be seen from Figure 7, the time advantage of the algorithm in this paper is relatively obvious, and the delivery time is relatively stable. The traditional ant algorithm has a single route, large time fluctuation, and poor antirisk ability. The delivery time of the driver experience method is also unstable. The driver mainly selects the route based on personal experience, and the delivery is relatively stable, but the route is not optimal. The traffic grade data between 5 a.m. and 22 p.m. of a day are randomly selected to build a time-sharing traffic network. The genetic algorithm, traditional ant algorithm, and heterogeneous neural network algorithm of logistics allocation system are used for comparative experiments. The starting and ending points are determined every 1 hour (12 periods). The comparison results are shown in Figure 8.

Figure 8 shows the change of distribution time in a continuous period of time in a day. It can be seen that the distribution time changes at any time with obvious fluctuation. In this paper, based on the heterogeneous neural network algorithm of the logistics allocation system, the distribution time in a day is shorter than the traditional ant algorithm and genetic algorithm. It has more obvious advantages in rush hours. The change in distribution time also reflects the change in road conditions to a certain extent.

## 5. Conclusion

This paper explains the problem of logistics distribution path optimization, introduces the application of the evolutionary algorithm in path optimization in detail, analyses the problems of the traditional evolutionary algorithm in today's complex road conditions, analyses the technical advantages of deep learning, and puts forward solutions. Aiming at the problem that the traditional path optimization algorithm does not deal with or simply deals with the influencing factors of road conditions, and the optimization ability decreases in today's complex urban road conditions, a deep learning model is introduced to learn the traffic data and influencing factors of road conditions. Set up the framework of the deep learning model suitable for traffic data training, construct neurons, complete the training of the model by using the method of layer-by-layer training and gradient descent, give the evaluation standard of the prediction model, and verify it in the test. The innovation of this paper is to introduce the heterogeneous neural network into the path optimization problem, solve the problem of weak practical application of traditional algorithms, and provide a new idea to solve the problem of logistics distribution path optimization. The disadvantage of this paper is that after the introduction of the graph neural network, the complexity and parameters of the model have increased a lot. Therefore, in order to make the model converge, more simulation data and greater computational performance are needed, which brings serious challenges to the applications with high computational efficiency. In the future, we will combine the changes in logistics distribution mode, make accurate planning and arrangement, and make further research on the efficient use of transportation distribution resources.

## Figures and Tables

**Figure 1:** Basic process of logistics distribution.

**Figure 2:** Flow chart of heterogeneous neural network path distribution.

**Figure 3:** Speed curve of roads and vehicles. (a) Road condition curve of traffic section; (b) curve of vehicle running speed.

**Figure 4:** Performance comparison of two methods. (a) *P* = 120, *S* = 120, *Z* = 120; (b) *P* = 240, *S* = 120, *Z* = 120; (c) *P* = 400, *S* = 120, *Z* = 120; (d) *P* = 500, *S* = 200, *Z* = 200.

**Figure 5:** The comparison between proposed method and traditional method.

**Figure 6:** Accuracy under different road conditions. (a) Forecast of working days; (b) forecast of working days; (c) accuracy of weekend forecast.

**Figure 7:** Distribution time chart of different methods.

**Figure 8:** Comparison chart of delivery time.

## Data Availability

All data, models, and code generated or used during the study appear in the submitted manuscript.
